The article "Case Report: Response to Almonertinib in a Patient With Metastatic NSCLC Resistant to Osimertinib due to Acquired EGFR L718Q Mutation" was published in 2021. Journal: Front Pharmacol.

# Case Report: Response to Almonertinib in a Patient With Metastatic NSCLC Resistant to Osimertinib due to Acquired EGFR L718Q Mutation

**DOI:** 10.3389/fphar.2021.731895

**Published:** 2021-12-20

**Authors:** Gang Shen, Lei Shi, Xin Tian, Depei Huang, Hao Chen, Chan Gao, Xudong Shen, Hushan Zhang

**Affiliations:** ^1^ Department of Thoracic Oncology, The Second Affiliated Hospital of Zunyi Medical University, Zunyi, China; ^2^ Department of Head and Neck Oncology, The Second Affiliated Hospital of Zunyi Medical University, Zunyi, China; ^3^ The Medical Department, 3D Medicines Inc., Shanghai, China; ^4^ The Bioinformatics Department, 3D Medicines Inc., Shanghai, China

**Keywords:** NSCLC-lung adenocarcinoma-EGFR-ALK-BRAF-KRAS-RET-MET-PD-L1-ROS1., EGFR, TKI-tyrosine kinase inhibitor, almonertinib, L718Q

## Abstract

Osimertinib shows strong clinical activity in first- and second-line treatment of nonsmall-cell lung cancer (NSCLC) patients with epidermal growth factor receptor (EGFR) mutations, especially EGFR T790M. However, when patients develop resistance, there is currently no definite postosimertinib treatment option. Herein, we report a patient with metastatic NSCLC who benefited from almonertinib after developing resistance to osimertinib.

## Introduction

EGFR is one of the four HER family receptor members, and the EGFR gene is an important oncogene in NSCLC. Blocking EGFR by specific TKIs through competitive binding with the EGFR binding region can inhibit EGFR activation and its downstream signaling pathways, with significant antitumor effects in NSCLC. EGFR TKIs such as gefitinib, erlotinib, afatinib, icotinib and third-generation TKIs such as osimertinib have been approved as standard care for NSCLC patients with mutations in the EGFR tyrosine kinase domain (TKD). However, acquired resistance almost inevitably develops after 9–15 months of treatment. Several mechanisms of acquired resistance have been demonstrated, including secondary EGFR mutations and mutations in bypass signaling pathways (Liu et al., 2017; Wu and Shih, 2018). The T790M mutation, involving substitution of threonine to methionine at amino acid 790, is the most common mechanism of resistance to first- and second-line EGFR TKI treatment. Osimertinib, currently approved as standard first-line treatment for NSCLC patients carrying EGFR mutations, also shows good activity for NSCLC patients with EGFR T790M mutants (Remon et al., 2018). Unfortunately, these patients, even those with EGFR T790M mutations, also eventually develop acquired resistance to osimertinib. The mechanisms reported include activating mutations in the bypass signaling pathway, loss of the T790M mutation, histological transformation, and acquisition of the EGFR C797S or EGFR L718Q mutation (Ma et al., 2019; Taniguchi et al., 2019; Mu et al., 2020). Overcoming drug resistance is a clinical problem that needs to be solved urgently, but there is no clear and solid strategy to date. Some alternatives for overcoming resistance to osimertinib have recently been reported, such as osimertinib, bevacizumab, and brigatinib combination therapy and brigatinib (Uchibori et al., 2017; Zhao et al., 2018; Shaikh et al., 2021). Based on a phase 2 expansion study of a phase 1/2 trial, the third-generation EGFR inhibitor almonertinib was approved in China in March 2020 for the treatment of advanced EGFR T790M-positive NSCLC (Yang et al., 2020; Nagasaka et al., 2021). Recent studies report that almonertinib has a good safety profile, with the parent drug as its main circulating component, and pharmacokinetic studies in a mouse model demonstrate a good ability of almonertinib to cross the blood–brain barrier (Zhang et al., 2021; Zhou et al., 2021). Herein, we present a case of resistance to osimertinib due to acquired EGFR L718Q mutation and subsequent response to almonertinib.

### Case Presentation

A 45-year-old Chinese woman was admitted to the Affiliated Hospital of Zunyi Medical University for comprehensive treatment of metastatic NSCLC. She underwent thoracoscopic right middle and lower lobectomy, partial left atrial resection, pericardiotomy, and lymph node dissection on November 21, 2017, with a confirmed histopathological diagnosis of stage ⅢC adenocarcinoma of the right middle lobe (pT4N3M0) **(** Figures 1A,B **)**. Postoperative diagnosis showed no tumor involvement in the parenchyma of the right lower lobe but cancer infiltration in the left atrial wall and left parabronchial bronchi; metastasis was detected in some mediastinal lymph nodes. The patient was found to carry an *EGFR* exon 19 deletion mutation by analysis of tissue specimens using next-generation sequencing (NGS) (Figure 1C). She received icotinib (125 mg/d, tid) treatment (Figure 2A). Eight months after icotinib treatment, CT showed metastases in the liver. Previous studies have demonstrated that patients develop resistance after a median of 10 months of EGFR TKI treatment (Wu and Shih, 2018). Based on this situation, icotinib was discontinued. Chemotherapy was performed for 24 days, and computed tomography (CT) revealed thoracic spine metastasis, suggestive of prior treatment failure. She then began to receive icotinib combined with bevacizumab, which was switched to chemotherapy 6 months later due to severe bone marrow suppression. A CT scan at that time showed progressive disease (PD), and analysis of circulating tumor DNA (ctDNA) revealed the *EGFR* T790M mutation (Figure 2B, 1D). She received osimertinib (80 mg, orally once daily) for 8 months, and then bevacizumab was added due to the progression of bone metastases. Eight months later, she was again found to have PD. Analysis of ctDNA showed the occurrence of *EGFR* L718Q **(** Figure 1E **)** and PLEKHH2-ALK fusions in addition to *EGF*R T790M. Therefore, osimertinib combined with erlotinib (150 mg, orally once daily) was initiated. Two weeks later, treatment was switched to crizotinib (250 mg twice daily) due to adverse events. One month later, the patient experienced dizziness, headache, and apathy. CT showed metastases in the bilateral parietal and left cerebellar regions and enlargement of the metastases in the liver **(** Figure 2B **)**. Crizotinib was discontinued. The patient could not tolerate brain radiotherapy and thus was given almonertinib (110 mg, orally once daily), and she showed a clinical response to almonertinib that lasted more than 2 months. Overall, her symptoms of dizziness, headache relieved, and mental state improved significantly at 1 week after almonertinib was initiated, and her Karnofsky score increased from 20 to 70. A CT scan two and a half months after almonertinib treatment initiation showed that both the liver and lung metastases were stable **(** Figure 2B **)**. Four months after almonertinib therapy, she was discharged from the hospital, though almonertinib was discontinued because of serious electrolyte disorders and heart failure.

**FIGURE 1:** Pathological diagnosis and molecular diagnosis. **(A,B)**, tumor specimen was applied to apex of right lung with a pathological diagnosis of lung adenocarcinoma (hematoxylin-eosin staining: 100x and 200x). **(C)**, Three-dimensional structure of EGFR protein with L718Q mutation predicted by MODELLER. Yellow represent structure of EGFR T790M, blue represent EGFR L718Q mutation, green represent TKI, and red circle present site of L718Q mutation. **(D–F)**, the mutations of EGFR were analyzed through NGS in a laboratory accredited by the College of American Pathologists (CAP) and Clinical Laboratory Improvement Amendment (CLIA) (3D Medicines Inc., Shanghai, China).

**FIGURE 2:** Acquired resistance to osimertinib and response to almonertinib. **(A)**, the various treatments the patient received and the duration of the various treatments. **(B)**, images of the patient’s metastatic lung, liver and brain disease.

## Discussion

Despite the robust efficacy of osimertinib, resistance to this drug is inevitable due to the lack of postosimertinib options (Leonetti et al., 2019). Mutation at EGFR L718 are responsible for osimertinib resistance *in vitro* and *in vivo*, and the amino acid is most frequently substituted with glutamine. This has recently been shown to be a mechanism of resistance to osimertinib, but few therapies can effectively overcome it (Yang et al., 2018; Leonetti et al., 2019). In the crystal structure of osimertinib in complex with EGFR, L718 is in direct contact with the aniline ring. Thus, the L718Q mutation may mediate drug resistance through steric hindrance and influence drug binding; that is, the glutamine side chain at position 718 is expected to sterically interfere with the position of osimertinib, reducing the efficiency of covalent bond formation (Yosaatmadja et al., 2015; Bersanelli et al., 2016). We used MODELLER, a computational protein structure modeling (Webb and Sali, 2016) technique, to predict the three-dimensional structure of the EGFR protein with the L718Q mutation, and the predicted structure is supported by the above theory that mutation of *EGFR* L718Q may affect binding between osimertinib and EGFR-TKD (Figure 1F). Amino acid 718 is found inside the p-loop of the EGFR TKD, which interacts with the aniline ring of osimertinib. According to the predicted model, mutation of this residue may cause spatial restriction and prevent osimertinib from binding to EGFR, that is, cause resistance to the drug. Despite some case reports that patients carrying the *EGFR* L718Q mutation might respond to afatinib (Starrett et al., 2020), there are no feasible and solid strategies available for overcoming acquired resistance to osimertinib caused by *EGFR* L718Q, especially with *EGFR* T790M and L718Q comutation (Shaikh et al., 2021). In fact, previous case reports and *in vitro* studies have revealed that afatinib only exhibits an inhibitory effect on phosphorylation in the presence of *EGFR* L858R + L718V/Q comutation (Starrett et al., 2020). Although our case involved *EGFR* L718Q in addition to the T790M mutation, resistance to osimertinib had already emerged.

The safety and efficacy of almonertinib (HS-10296), a novel, third-generation epidermal growth factor receptor tyrosine kinase inhibitor (EGFR-TKI), was evaluated in a phase I trial including patients with locally advanced or metastatic EGFR-mutated nonsmall-cell lung cancer (NSCLC) whose disease had progressed after prior EGFR TKI therapy (Yang et al., 2020). As previously reported, the main adverse events of all grades with almonertinib treatment of NSCLC patients were rash, pruritis, leukopenia, and increases in creatinine phosphokinase, alanine aminotransferase and aspartate aminotransferase, with increases in creatinine phosphokinase and alanine aminotransferase being the most common grade 3–4 adverse events (Yang et al., 2020; Nagasaka et al., 2021). In our case, unfortunately, almonertinib treatment ultimately discontinued due to serious electrolyte disorders and heart failure. However, according to previous evidence, electrolyte disorders and heart failure may be associated with accumulation of toxicity due to previous multiline treatment, whereby the physical constitution becomes very poor, rather than being due to almonertinib treatment.

## Conclusion

We report an NSCLC patient with metastasis and osimertinib resistance who benefitted from almonertinib. First, this case confirms resistance to osimertinib caused by the L718Q mutation. In addition, this case suggests that almonertinib has the potential to overcome resistance to osimertinib associated with the L718Q mutation and that NGS can be used as an effective method for EGFR mutation analysis. It may be very meaningful that NGS detection accompanies systemic treatment of advanced NSCLC patients or is used for monitoring NSCLC patients postoperatively. As more evidence accumulates, NGS accompanying monitoring may become a powerful clinical diagnosis and treatment tool.

## Data Availability

The original contributions presented in the study are included in the article/Supplementary Material, further inquiries can be directed to the corresponding author.

## Abbreviations

EGFR, Epidermal Growth Factor Receptor; NGS, next-generation sequencing; NSCLC, Non-small cell lung cancer.
